RETRACTED

# Fetal Congenital Cardiac and Vascular Disorders Associated with Sertraline Treatment during Pregnancy: Analysis of FAERS Data

**DOI:** 10.1155/2022/9914931

**Published:** 2022-07-13

**Authors:** Fanzhen Hong, Jianqing Qiu, Shanshan Zhang, Lei Zhang

**Affiliations:** ^1^Department of Obstetrics, The Second Hospital, Cheeloo College of Medicine, Shandong University, No. 247 Beiyuan Road, Tianqiao District, Jinan, Shandong Province, China; ^2^Department of Obstetrics, Jining First People's Hospital, No. 6 Jiankang Road, Rencheng District, Jining, Shandong Province, China

## Abstract

**Objective:**

Sertraline is one of the most commonly used antidepressants worldwide and is one of the first-choice treatments for depression during pregnancy. This study is aimed at testing the possible association between sertraline intrauterine exposure and congenital cardiac and vascular disorder occurrences by assessing the publicly available US Food and Drug Administration Adverse Event Reporting System (FAERS).

**Methods:**

Disproportionality analysis and Bayesian analysis were used to mine FAERS for suspected congenital cardiac and vascular disorder data for sertraline intrauterine exposure from the first quarter of 2004 to the second quarter of 2021.

**Results:**

Among the 914 cases of sertraline used with congenital cardiovascular disease in the FAERS database, the reporting areas were mainly in the United States and Europe. The number of adverse events reported every year since 2004 has no many differences. Congenital anomalies are the most frequently reported serious clinical outcome. Among the 69 positive signals detected from 914 cases, 31 were invalid signals, and 38 were valid signals according to criteria. The most common ones are heart disease congenital, atrial septal defect, ventricular septal defect, patent ductus arteriosus, and persistent fetal circulation.

**Conclusions:**

Mining FAERS data can analyze and study the adverse reactions of sertraline in a more comprehensive and in-depth manner, thereby effectively reducing the risk of clinical medication.

## 1. Introduction

The prevalence rate of depression during pregnancy is high, ranging from 7% to 20% [1]. Depression during pregnancy is associated with smoking, maternal malnutrition, alcohol, insufficient weight gain and other substance intake, and increased risk of postpartum depression [2]. Nonpharmacological interventions are more suitable for mild-to-moderate depression, while antidepressant prescribing is preferable for severe depression or when other treatments are unavailable or ineffective [3]. Deciding whether to stop, change, or start antidepressants during pregnancy requires weighing the treatment-related maternal and infant risks with untreated depression-related risks. The widespread use of antidepressants during pregnancy makes it essential to understand the safety and the risk of adverse outcomes in the fetus.

RETRACTED

Selective serotonin reuptake inhibitors (SSRIs) are considered as the most prescribed antidepressants during pregnancy because of its wealth and reassuring of data [4]. Approximately 63% to 85% of pregnant women who exposed to antidepressants are treated with SSRI [5]. Among the SSRIs, sertraline is one of the most commonly used antidepressants worldwide and is one of the first-choice treatments for depression during pregnancy [6, 7]. SSRIs are believed to be effective in treating psychiatric disorders by increasing the synaptic bioavailability of the neurotransmitter serotonin (5-HT) [8]. 5-HT easily crosses the placenta and plays a role in cardiac morphogenesis during endocardial cushion formation, which may cause heart malformations [9]. In addition, Sari and Zhou suggested that serotonin can promote the proliferation of fetal heart cells, and abnormal levels of serotonin or abuse of serotonin uptake blockers may alter heart development [10]. Several studies [11, 12] have shown that sertraline increases the risk of cardiovascular-related malformations in infants, while other studies [13, 14] found no correlation at all. Because studies of antidepressants in pregnancy are usually not random, it is often difficult to determine whether the adverse results associated with antidepressants are related to the drug itself and other confounding exposures (such as alcohol, smoking, drug abuse, nutrition, and other drugs). Considering that the scope of application of sertraline has been expanded to special populations such as pregnant women, it is necessary to dig deeper into its adverse reaction signals to avoid drug risks and ensure drug safety.

Some countries or organizations have established pharmacovigilance systems, such as the US Food and Drug Administration (FDA), European Medicines Agency (EMA), and the World Health Organization (WHO), for adverse drug reaction (ADR) monitoring. The FDA's Adverse Event Reporting System (FAERS) is the largest repository of passively reported adverse drug events worldwide [15]. Given the inconsistency of previous results, as well as to provide the best estimates of the effect of sertraline usage during pregnancy, we performed a real-world analysis of FAERS to investigate the association between sertraline treatment and congenital cardiac and vascular disorders, with a view to revealing the regularity of sertraline adverse events, and for the control and management of sertraline safety risks, providing reference for clinical rational use of sertraline.

RETRACTED

## 2. Material and Methods

### 2.1. Data Source

A retrospective pharmacovigilance study was performed using data from FAERS database covering period from the first quarter of 2004 to the second quarter of 2021. FAERS is a spontaneous reporting system (SRS) that contains adverse event reports, medication error reports, and product quality complaints resulting in adverse events submitted to FDA by healthcare professionals, consumers, manufacturers, and patients. The database contains demographic information, drug information, and reaction information. Each report has a primary suspected drug with one or more adverse drug reactions (ADR) and may include other drugs taken by the patient [16].

The ASCII data files of the FAERS contain demographic and administrative information (DEMO), drug information (DRUG), adverse events (REAC), patient outcomes (OUTC), report sources (RPSR), therapy start dates and end dates for reported drugs (THER), and indications for use (INDI).

A total of 15881123 reports were retrieved from the FAERS. A deduplication procedure was performed according to the FDA's recommendations to select the latest FDA_DT with the same CASEID and select the higher PRIMARYID when CASEID and FDA_DT are both the same, resulting in a reduction in the number of reports to 13327865. On the basis of the PRIMARYID of the deduplicated DEMO, DRUG and REAC were both deduplicated as well.

### 2.2. Data Mining

FAERS data requires substantial curated cleaning and normalizing before they can be used appropriately; otherwise, data can have material impact on analysis results. We used Python (version 3.8) and PostgreSQL (version 12) to deal with cleaning and normalizing process which includes merging data, deduplicating records, applying standardized vocabularies with drug names mapped to RxNorm concepts and indications and outcomes mapped to SNOMED-CT concepts, and normalizing reaction to MedDRA (version 24.0) concepts and used the R software (version 4.1.0) to statistical compute drug-reaction signals.  Figure 1 presents main steps.

### 2.3. Statistical Analysis

“Sertraline” was chosen as the drug name with a reported role code “PS” (primary suspect drug) [17] and reactions with the MedDRA SOC term “congenital, familial, and genetic disorders” (MedDRA code: 10010331) from DRUG_REACTION PAIRS to be evaluated. In total, 127 drug-reaction pairs were retrieved.

Both disproportionality analysis and Bayesian analysis applied with the use of the reporting odds ratio (ROR), proportional reporting ratio (PRR), Bayesian confidence propagation neural network (BCPNN), and multi-item gamma Poisson shrinker (MGPS) algorithms were used to investigate the potential signals between the drug and the specific adverse event of interest. The equations and criteria for the four algorithms above [18–25] are demonstrated in Table 1. One of the four algorithms meet the criteria should be considered as a positive signal.

RETRACTED

### 2.4. Compliance with Ethics Guidelines

All procedures performed in this study involving human participants were in accordance with the 1964 Helsinki declaration. This study was exempted from approval by the ethics committee of the Second Hospital of Shandong University.

## 3. Results

In total, 914 cases of intrauterine sertraline exposure with fetal congenital cardiovascular disease were identified in the FAERS database. Of these events, 43% occurred in male offspring, 42.23% occurred in female offspring, and 14.77% of the events were gender unknown (Table 2). It noted that a case may have multiple clinical outcomes. The proportion of males and females in offspring of 914 cases is balanced, consistent with the results of previous studies, and there is no obvious gender difference in offspring.

The number of adverse events reported every year since 2004 has no many differences, which demonstrates the stable safety of sertraline for a long period (Table 2). The majority of adverse events came from the Americas (724 (79.3%)) (Table 2). In most reports, congenital anomalies (774, 41.21%) are the most frequently reported serious clinical outcome, and other serious events (major medical events) or hospitalizations (initial or long-term) are 664 (35.36%) and 220 (11.71%), respectively. Since the adverse reactions in this study are all associated with the congenital diseases of offspring after intrauterine sertraline exposure, the patient's outcome is described from the babies born in the population identified in this study and related to congenital disease characteristics.

Among the 69 positive signals detected from 914 cases, 31 were invalid signals, and 38 were valid signals according to criteria. The most common ones are heart disease congenital (PT: 10019273), atrial septal defect (PT: 10003664), ventricular septal defect (PT: 10047298), patent ductus arteriosus (PT: 10034130), and persistent fetal circulation (PT: 10034708) (Table 3).

The most common clinical indications for sertraline in the report were depression 355 (51.52%) and anxiety 136 (19.74%), which are consistent with the indications of sertraline (Table 4). Since the disease in this study is a congenital disease, all reports occurred in infants and young children (<36 M) (Table 5). The five most common adverse events of sertraline were atrial septal defect (PT: 10003664), heart disease congenital (PT: 10019273), ventricular septal defect (PT: 10047298), patent ductus arteriosus (PT: 10034130), and persistent fetal circulation (PT: 10034708).

RETRACTED

## 4. Discussion

SSRI may be associated with an increased risk for birth defects or congenital heart defects overall [1, 12, 26, 27], although findings are occasionally mixed. In this study, we focused on the risks of sertraline medication to the fetus related to the fetal congenital heart diseases during pregnancy. The adverse reaction signals detected based on the FAERS database are quite different from the common adverse reactions of fetus in sertraline's instructions. The very common adverse reactions associated with fetus exposed to sertraline during pregnancy in the instructions dyspnea, cyanosis, apnea, seizures, unstable body temperature, difficulty feeding, vomiting, hypoglycemia, hypotonia, increased muscle tone, tendon hyperreflexia, tremor, nervousness, irritability, and constant crying noise. The side effects of strong sertraline signal related to fetal safety are congenital heart and vascular disorders, including corrected transposition of great vessels, newborn persistent pulmonary hypertension, shone complex, congenital mitral valve stenosis, congenital tricuspid valve stenosis, congenital coronary artery malformation, and congenital aortic valve stenosis, from the results of this study. These are different from the common adverse reactions of sertraline given in the instructions, indicating that the discovery of adverse reactions related to sertraline therapy during pregnancy and fetal congenital diseases is worthy of additional attention in clinical prescription and adequate measurement of the benefits and risks of medication during pregnancy. Due to ethical restrictions, there is currently no high-quality prospective randomized double-blind controlled study on the relationship between intrauterine exposure to sertraline and abnormal development of offspring in pregnant women. Previous population-based cohort studies have shown that utero exposure of sertraline in the first trimester is significantly associated with fetal atrial or ventricular defects [28], and a meta-analysis showed that the intrauterine exposure of sertraline in the first trimester was significantly related to the offspring's atrial septal defect and/or ventricular septal defect [12]. Our finding is also consistent with above researches. In our study, there are totally 914 cases with fetal congenital heart diseases reported in the database which are related to sertraline intrauterine exposure. Among these cases, 127 cases are reported as atrial septal defect, and 99 cases are reported as ventricular septal defect, which are all strongly related with utero exposure of sertraline during pregnancy.

RETRACTED

Embryonic development is a complex process; it is commonly accepted that the first trimester of pregnancy is a key period in fetal development (i.e., sensitive period to teratogenic agent). Therefore, studies in the literature have explored the effects of intrauterine exposure of sertraline in the first trimester on the fetus. However, in these studies, the number of malformations after exposure is small, which is related to the lower incidence of fetal malformations. The number of positive cases may cause deviations in the results. FAERS database collects the global adverse drug reaction reporting data, which has a higher population base. We analyzed the FAERS database and obtained 914 cases of fetal heart development related adverse reactions after sertraline exposure and obtained 69 adverse reaction entries through statistical analysis, which obtained more positive results compared with the previous literature. The vast majority of the 69 adverse reactions significantly related to sertraline intrauterine exposure were structural abnormalities of fetal cardiovascular system, of which 38 were strongly significantly associated with, except that “trisomy 21” was not related to cardiovascular system; the other 31 were adverse reactions of cardiovascular system, which were structural malformations. The above results from the real-world analysis of FAERS have also been more accurately verified by echocardiography in the studies performed by Ansah et al. [29] and Kolding et al. [30]. The cardiac function of fetuses without cardiac structural malformation exposed to sertraline was evaluated; the results of both studies showed that sertraline intrauterine exposure did not cause changes in fetal cardiac function under the premise of no structural malformations. However, the ventricular size of the sertraline intrauterine exposure group was significantly smaller than that of the control group, which suggested that sertraline has a specific effect on the structural development of fetal heart. Animal experiments also support the effect of sertraline exposure on cardiac development of offspring [31]. In the results of this study, we mined the types of fetal malformations related to sertraline intrauterine exposure based on larger population data, which added new evidence for specific fetal cardiovascular abnormalities caused by sertraline intrauterine exposure.

In sertraline's instructions, persistent pulmonary hypertension (PPHN) is the only clearly stated description of adverse reactions of fetal malformations; the relationship between it and SSRIs has been discussed in related studies [32]. Masarwa et al. [33] conducted a systematic review, estimating the risks of maternal exposure to SSRI, SNRI, and PPHN, and the results indicated that exposure to SSRI and/or SNRI at any stage of pregnancy significantly increased the risk of PPHN (OR = 1.82; 95% CI: 1.31~2.54). Sertraline's instruction also mentions that exposure of infants to SSRIs in late pregnancy may increase the risk of persistent pulmonary hypertension (PPHN) in newborns. In addition, pregnant women using SSRIs tend to be older, more likely to smoke, higher body mass index, and higher frequency of caesarean section [34], which are potential risk factors for PPHN. Although there is no conclusive evidence for the risk of PPHN after exposure to SSRIs during pregnancy, this study, based on the evidence from the FAERS database, confirms the connection between sertraline and PPHN from another perspective, providing evidence-based on the real world. However, the number of reported cases of PPHN in the adverse reactions we analyzed only ranked 14th; the results of this study show that maternal sertraline application during pregnancy has more potential risk of cardiovascular malformations in offspring. Moreover, there is no obvious downward trend in the number of adverse reaction cases reported every year, suggesting that sertraline still has a relatively stable clinical application in pregnant women. Testing institutions and clinical practice should be vigilant, and there should be more perfect drug instructions to remind doctors and patients to fully evaluate the risks and benefits before medication.

RETRACTED

In the results of this study, one of the items of abnormal offspring development caused by sertraline intrauterine exposure is corrected transposition of great vessels. Corrected transposition of great vessels is a rare complex congenital heart disease often accompanied by ventricular septal defect, pulmonary artery stenosis or atresia, Ebstein-like malformation of the tricuspid valve, and median heart, and is worth noting because it has the highest reporting odds ratio of ROR, PRR, and EBGM. Moreover, corrected transposition of great vessels has not been noticed in previous sertraline-related studies. Moreover, due to the highest reporting odds ratio of the corrected transposition of great vessels but the low frequency, there may be statistical deviations. The pathogenesis of corrected transposition of great vessels is still unclear; the specific mechanism of sertraline interfering with fetal programming in uterus requires further experimental research.

Among the fetal adverse reactions significantly related to sertraline exposure analyzed in this study, three terms are more interesting, namely, trisomy 21, trisomy 18, and trisomy 13, of which trisomy 21 is strongly related. At present, no reports and studies have been retrieved about the intrauterine exposure of sertraline during pregnancy and the chromosomal abnormalities of the offspring. However, with the existence of 5-HT and its receptor in female reproductive system and subsequent functional researches, 5-HT was believed to play an important role in egg maturation and early embryonic development [35]. In animal models, SSRI drugs can cause abnormal follicular development by acting on ovaries [36]. Therefore, the effect of sertraline on chromosome abnormalities in offspring may be related to this. In the correlation analysis between chromosomal abnormalities and sertraline intrauterine exposure, ROR, PRR, BCPNN, and EBGM showed statistical differences; however, we note that the reported number of trisomy 21 cases is 8, trisomy 18 cases are 2, and trisomy 13 cases are 1; a small number of cases may also affect the analysis results. In brief, this study found that there was a significant correlation between intrauterine sertraline exposure during pregnancy and the triploidy of offspring trisomy 21, trisomy 18, and trisomy 13, but more rigorous prospective cohort studies were needed.

RETRACTED

The specific mechanism of fetal cardiovascular malformation caused by sertraline intrauterine exposure is not clear. In this study and previous literature, the gender of offspring did not show a significant correlation with cardiovascular malformations in sertraline exposed cases, suggesting that gender has nothing to do with the incidence [28]. Animal experiments showed that sertraline intrauterine exposure resulted in a significant decrease in Akt phosphorylation, proliferation, and cardiocyte cross-sectional area of offspring cardiomyocytes, resulting in a dose-dependent effect on cardiac structure and function [31]. Current studies have found that 5-HT is not only a neurotransmitter but also an important regulator in the biological process of embryonic heart development and participates in the regulation of key events in heart development [9]. Previous studies have confirmed that the concentration of sertraline in amniotic fluid is significantly correlated with the maternal intake dose, suggesting that the maternal intake of sertraline may spread to the fetal circulation through the placenta and then interfere with the embryonic heart development process through the above mechanisms [37]. Currently, the mechanism of 5-HT in the development of human embryonic cardiovascular system has not been clarified; an in-depth mechanism study should be carried out to provide more evidence for the safety of drugs during pregnancy.

RETRACTED

Further excavation of the FAERS database can expand new ideas for evaluating the safety of drugs used during pregnancy and is a research method that is worthy of further in-depth development. But this method also has limitations. First, because FAERS data is a voluntary report, including public reports, there are problems such as underreporting, selective reporting, and lack of information. In addition, although the analysis shows that there is a statistical correlation between the drug and the adverse event, the actual causality still needs further verification. In addition, most of the FAERS data come from European and American populations and relatively few Asian populations.

## 5. Conclusion

In this study, ADR signal detection is carried out through the FAERS database; a comprehensive and in-depth analysis indicated that the maternal application of sertraline during pregnancy has a significant association with cardiac abnormalities of offspring. This result provides new supplements for the related adverse reactions in the instructions and also provides an objective basis for clinical safe medication. At the same time, the detection of adverse reaction signals should also rely on large, well-organized epidemiologic studies to obtain relatively sufficient evidence.

## Figures and Tables

**Figure 1:** Main steps of process.

**Table 1:** Summary of major algorithms and criteria used for signal detection.

Algorithms	Equation	Criteria
ROR	$\text{ROR}=\frac{ad}{bc}$	ROR ≥ 1; CI025 ≥ 1
	$95\%\text{CI}=e^{\ln\left(\text{ROR}\right)\pm 1.96\sqrt{\frac{1}{a}+\frac{1}{b}+\frac{1}{c}+\frac{1}{d}}}$	
PRR	$\text{PRR}=\frac{a\left(c+d\right)}{c\left(a+b\right)}$	PRR ≥ 2; *χ*^2^ ≥ 4; *a* ≥ 3
	$95\%\text{CI}=e^{\ln\left(\text{PRR}\right)\pm 1.96\sqrt{\frac{1}{a}-\frac{1}{a+b}+\frac{1}{c}+\frac{1}{c+d}}}$	
	$\chi^{2}=\sum \frac{{\left(O-E\right)}^{2}}{E};\left(O=a,E=\frac{\left(a+b\right)\left(a+c\right)}{a+b+c+d}\right)$	
BCPNN	IC = log_2_*a*(*a* + *b* + *c* + *d*)(*a* + *c*)(*a* + *b*)	IC25 − 2sd > 0
	$95\%\text{CI}=e^{\ln\left(\text{IC}\right)\pm 1.96\sqrt{\frac{1}{a}+\frac{1}{b}+\frac{1}{c}+\frac{1}{d}}}$	
MGPS	$\text{EBGM}=\frac{a\left(a+b+c+d\right)\left(a+b\right)}{a+c}$	EBGM05 ≥ 2
	$95\%\text{CI}=e^{\ln\left(\text{EBGM}\right)\pm 1.96\sqrt{\frac{1}{a}+\frac{1}{b}+\frac{1}{c}+\frac{1}{d}}}$	

ROR: reporting odds ratio; PRR: proportional reporting ratio; BCPNN: Bayesian confidence propagation neural network; MGPS: multi-item gamma Poisson shrinker.

**Table 2:** Characteristics of reports associated with sertraline.

	Reports no.	%
Reporting region		
Europe	145	15.86%
Oceania	2	0.22%
Americas	729	79.76%
Asia	37	4.05%
Africa	1	0.11%
Reported year		
2004 and before	224	24.42%
2005	47	5.15%
2006	58	6.35%
2007	58	6.35%
2008	60	6.57%
2009	55	6.02%
2010	78	8.54%
2011	68	7.45%
2012	44	4.82%
2013	11	1.2%
2014	35	3.83%
2015	33	3.61%
2016	49	5.37%
2017	25	2.74%
2018	10	1.1%
2019	31	3.4%
2020	20	2.19%
2021Q1Q2	8	0.88%
Gender		
Female	386	42.23%
Male	393	43%
Unknown	135	14.77%
Outcome		
Congenital anomaly	774	41.21%
Death	67	3.57%
Disability	21	1.12%
Hospitalization—initial or prolonged	220	11.71%
Life-threatening	124	6.6%
Other serious (important medical event)	664	35.36%
Required intervention to prevent permanent impairment/damage	8	0.43%

RETRACTED

**Table 3:** Signal detection for sertraline-associated congenital cardiovascular disease in the FAERS database.

Reaction (PT code)	Case	ROR (95% two-sided CI)	PRR (95% two-sided CI, *χ*^2^)	BCPNN (IC-2SD)	EBGM (90% two-sided CI)	
Heart disease congenital (10019273)	128	22.6 (18.88, 27.06)	22.56 (22.38, 22.74, 2429.61)	4.19 (4.12)	21.02 (20.87, 21.17)	*P* ^∗^
Atrial septal defect (10003664)	127	15.63 (13.07, 18.69)	15.6 (15.42, 15.78, 1634.23)	3.74 (3.69)	14.86 (14.71, 15.01)	*P* ^∗^
Ventricular septal defect (10047298)	99	16.12 (13.17, 19.74)	16.1 (15.90, 16.30, 1315.07)	3.74 (3.68)	15.32 (15.15, 15.49)	*P* ^∗^
Patent ductus arteriosus (10034130)	72	19.15 (15.09, 24.31)	19.13 (18.89, 19.37, 1144.72)	3.87 (3.78)	18.02 (17.82, 18.22)	*P* ^∗^
Persistent fetal circulation (10034708)	34	37.82 (26.46, 54.06)	37.8 (37.45, 38.16, 1047.24)	4.12 (3.95)	33.62 (33.32, 33.92)	*P* ^∗^
Fallot's tetralogy (10016193)	30	20.42 (14.11, 29.57)	20.41 (20.04, 20.78, 499.97)	3.59 (3.46)	19.16 (18.85, 19.47)	*P* ^∗^
Transposition of the great vessels (10044443)	27	24.12 (16.29, 35.71)	24.11 (23.72, 24.50, 531.58)	3.66 (3.51)	22.36 (22.03, 22.69)	*P* ^∗^
Pulmonary valve stenosis congenital (10037451)	21	35.17 (22.37, 55.30)	35.16 (34.70, 35.61, 592.37)	3.72 (3.51)	31.52 (31.14, 31.89)	*P* ^∗^
Cardiac septal defect (10064021)	21	29.2 (18.65, 45.72)	29.19 (28.74, 29.64, 494.71)	3.62 (3.43)	26.65 (26.27, 27.02)	*P* ^∗^
Pulmonary artery stenosis congenital (10037339)	20	21.05 (13.37, 33.14)	21.05 (20.59, 21.50, 337.90)	3.38 (3.21)	19.71 (19.33, 20.09)	*P* ^∗^
Coarctation of the aorta (10009807)	19	14.11 (8.90, 22.35)	14.1 (13.64, 14.56, 208.35)	3.05 (2.91)	13.5 (13.12, 13.89)	*P* ^∗^
Hypoplastic left heart syndrome (10021076)	18	19.58 (12.15, 31.55)	19.57 (19.09, 20.05, 280.22)	3.26 (3.09)	18.41 (18.01, 18.81)	*P* ^∗^
Bicuspid aortic valve (10004552)	17	22.27 (13.60, 36.46)	22.26 (21.77, 22.76, 301.45)	3.3 (3.12)	20.77 (20.36, 21.18)	*P* ^∗^
Newborn persistent pulmonary hypertension (10053592)	15	176.83 (93.23, 335.42)	176.79 (176.15, 177.43, 1530.31)	3.81 (3.36)	110.87 (110.33, 111.40)	*P* ^∗^
Haemangioma congenital (10018818)	14	40.85 (23.36, 71.45)	40.84 (40.28, 41.40, 443.43)	3.43 (3.16)	35.99 (35.52, 36.46)	*P* ^∗^
Congenital cardiovascular anomaly (10061054)	14	8.72 (5.13, 14.84)	8.72 (8.19, 9.25, 85.58)	2.5 (2.37)	8.5 (8.05, 8.94)	*P* ^∗^
Congenital heart valve disorder (10064086)	12	35.36 (19.43, 64.36)	35.36 (34.76, 35.96, 327.59)	3.23 (2.96)	31.68 (31.18, 32.18)	*P* ^∗^
Congenital aortic valve stenosis (10010371)	9	57.66 (28.22, 117.80)	57.65 (56.93, 58.36, 372.82)	3.07 (2.69)	48.38 (47.78, 48.98)	*P* ^∗^
Hypertrophic cardiomyopathy (10020871)	9	7.78 (4.01, 15.08)	7.78 (7.11, 8.44, 45.37)	2.19 (2.04)	7.6 (7.05, 8.16)	*P* ^∗^
Congenital coronary artery malformation (10061060)	8	58.94 (27.59, 125.92)	58.93 (58.17, 59.69, 332.75)	2.95 (2.54)	49.27 (48.64, 49.91)	*P* ^∗^
Trisomy 21 (10044688)	8	5.12 (2.55, 10.31)	5.12 (4.43, 5.82, 22.19)	1.8 (1.67)	5.05 (4.47, 5.64)	*P* ^∗^
Pulmonary artery atresia (10037337)	8	47.15 (22.35, 99.46)	47.14 (46.40, 47.89, 272.85)	2.91 (2.53)	40.78 (40.15, 41.40)	*P* ^∗^
Double outlet right ventricle (10013611)	7	18.42 (8.58, 39.53)	18.42 (17.65, 19.18, 92.68)	2.51 (2.24)	17.39 (16.75, 18.03)	*P* ^∗^
Shone complex (10066802)	6	104 (41.00, 263.80)	103.99 (103.06, 104.92, 379.20)	2.69 (2.11)	77.13 (76.35, 77.90)	*P* ^∗^
Aorta hypoplasia (10049209)	5	16.01 (6.51, 39.39)	16.01 (15.11, 16.91, 53.23)	2.17 (1.88)	15.24 (14.49, 15.99)	*P* ^∗^
Congenital mitral valve stenosis (10010548)	5	73.67 (27.65, 196.29)	73.66 (72.68, 74.64, 231.34)	2.46 (1.90)	59.13 (58.31, 59.95)	*P* ^∗^
Multiple cardiac defects (10028178)	5	22.32 (8.99, 55.41)	22.32 (21.41, 23.23, 75.82)	2.27 (1.93)	20.82 (20.06, 21.58)	*P* ^∗^
Anomalous pulmonary venous connection (10058079)	4	12.41 (4.56, 33.74)	12.41 (11.41, 13.41, 30.02)	1.9 (1.61)	11.95 (11.11, 12.78)	*P* ^∗^
Atrioventricular septal defect (10063836)	4	7.96 (2.95, 21.50)	7.96 (6.97, 8.96, 17.40)	1.72 (1.49)	7.78 (6.95, 8.61)	*P* ^∗^
Congenital aortic stenosis (10010369)	4	13.87 (5.09, 37.80)	13.87 (12.86, 14.87, 34.11)	1.94 (1.63)	13.29 (12.45, 14.13)	*P* ^∗^
Corrected transposition of great vessels (10011120)	4	589.33 (107.94, 3217.69)	589.29 (587.60, 590.99, 598.66)	2.29 (1.20)	197.1 (195.68, 198.52)	*P* ^∗^
Ventricular hypoplasia (10047296)	3	10.16 (3.21, 32.12)	10.16 (9.01, 11.31, 15.89)	1.61 (1.31)	9.85 (8.89, 10.82)	*P* ^∗^
Univentricular heart (10045545)	3	18.81 (5.85, 60.43)	18.81 (17.64, 19.97, 32.23)	1.77 (1.37)	17.74 (16.76, 18.72)	*P* ^∗^
Truncus arteriosus persistent (10044703)	3	23.89 (7.37, 77.49)	23.89 (22.71, 25.07, 41.47)	1.81 (1.36)	22.17 (21.19, 23.16)	*P* ^∗^
Congenital pulmonary artery anomaly (10061074)	3	19.22 (5.98, 61.79)	19.22 (18.05, 20.38, 32.99)	1.77 (1.37)	18.1 (17.12, 19.08)	*P* ^∗^
Congenital tricuspid valve stenosis (10010656)	3	73.67 (20.79, 261.06)	73.66 (72.40, 74.93, 118.64)	1.92 (1.20)	59.13 (58.07, 60.19)	*P* ^∗^
Congenital pulmonary valve atresia (10052644)	3	8.26 (2.62, 26.02)	8.26 (7.11, 9.41, 12.21)	1.54 (1.27)	8.06 (7.10, 9.02)	*P* ^∗^
Dextrocardia (10012592)	3	15.24 (4.78, 48.64)	15.24 (14.08, 16.40, 25.58)	1.73 (1.36)	14.54 (13.57, 15.51)	*P* ^∗^
Congenital pulmonary valve disorder (10061075)	2	15.93 (3.84, 66.09)	15.93 (14.50, 17.35, 14.24)	1.4 (0.95)	15.16 (13.97, 16.35)	*P*
Trisomy 18 (10053884)	2	5.12 (1.27, 20.74)	5.12 (3.73, 6.52, 3.09)	1.1 (0.83)	5.05 (3.88, 6.22)	*P*
Hypoplastic right heart syndrome (10064962)	2	8.93 (2.19, 36.46)	8.93 (7.52, 10.34, 7.04)	1.28 (0.93)	8.7 (7.52, 9.87)	*P*
Noonan syndrome (10029748)	2	39.29 (8.98, 171.81)	39.29 (37.81, 40.76, 36.31)	1.5 (0.82)	34.78 (33.55, 36.02)	*P*
Congenital arterial malformation (10062325)	2	11.56 (2.81, 47.47)	11.55 (10.14, 12.97, 9.76)	1.34 (0.95)	11.16 (9.97, 12.34)	*P*
Vascular malformation (10074979)	2	8.54 (2.09, 34.84)	8.54 (7.13, 9.95, 6.63)	1.27 (0.93)	8.33 (7.15, 9.50)	*P*
Right ventricle outflow tract obstruction (10064195)	2	14.03 (3.40, 57.97)	14.03 (12.61, 15.45, 12.31)	1.38 (0.95)	13.44 (12.25, 14.63)	*P*
Congenital aortic anomaly (10061052)	2	8.67 (2.12, 35.36)	8.67 (7.26, 10.07, 6.76)	1.27 (0.93)	8.45 (7.27, 9.62)	*P*
Congenital mitral valve incompetence (10010547)	2	13.7 (3.32, 56.58)	13.7 (12.29, 15.12, 11.98)	1.38 (0.95)	13.14 (11.95, 14.33)	*P*
Interruption of aortic arch (10022599)	2	22.67 (5.38, 95.50)	22.67 (21.23, 24.10, 20.92)	1.45 (0.91)	21.12 (19.91, 22.32)	*P*
Cor triatriatum (10010972)	1	49.11 (5.91, 407.93)	49.11 (46.99, 51.22, 9.62)	0.96 (-0.06)	42.24 (40.46, 44.01)	*P*
Digeorge's syndrome (10012979)	1	7.96 (1.09, 58.04)	7.96 (5.98, 9.95, 1.08)	0.82 (0.36)	7.78 (6.12, 9.44)	*P*
Heart block congenital (10019263)	1	10.91 (1.48, 80.31)	10.91 (8.92, 12.91, 1.74)	0.87 (0.33)	10.56 (8.89, 12.23)	*P*
Trisomy 13 (10044686)	1	5.56 (0.77, 40.20)	5.56 (3.58, 7.54, 0.55)	0.75 (0.36)	5.48 (3.82, 7.13)	*P*
Congenital aortic dilatation (10058150)	1	32.74 (4.15, 258.43)	32.74 (30.67, 34.80, 6.45)	0.95 (0.08)	29.56 (27.84, 31.29)	*P*
Persistent left superior vena cava (10064193)	1	8.42 (1.15, 61.45)	8.42 (6.43, 10.41, 1.18)	0.83 (0.36)	8.21 (6.55, 9.88)	*P*
Aorticopulmonary septal defect (10063732)	1	32.74 (4.15, 258.43)	32.74 (30.67, 34.80, 6.45)	0.95 (0.08)	29.56 (27.84, 31.29)	*P*
Malformation venous (10025532)	1	10.16 (1.38, 74.59)	10.16 (8.17, 12.15, 1.57)	0.86 (0.34)	9.85 (8.19, 11.52)	*P*
Ebstein's anomaly (10014075)	1	5.17 (0.72, 37.33)	5.17 (3.19, 7.15, 0.47)	0.74 (0.36)	5.1 (3.44, 6.75)	*P*
Fallot's pentalogy (10059205)	1	147.33 (13.36, 1624.84)	147.32 (144.92, 149.72, 23.73)	0.98 (-0.46)	98.55 (96.54, 100.56)	*P*
Ductus arteriosus stenosis fetal (10013808)	1	1.94 (0.27, 13.85)	1.94 (-0.03, 3.90, 0.00)	0.4 (0.16)	1.93 (0.29, 3.58)	*P*
Ductus arteriosus premature closure (10049996)	1	1.89 (0.26, 13.49)	1.89 (-0.08, 3.86, 0.00)	0.38 (0.15)	1.88 (0.24, 3.53)	*P*
Vacterl syndrome (10066022)	1	5.36 (0.74, 38.71)	5.36 (3.38, 7.33, 0.51)	0.75 (0.36)	5.28 (3.62, 6.93)	*P*
Congenital aortic atresia (10010368)	1	24.55 (3.19, 188.85)	24.55 (22.51, 26.59, 4.75)	0.93 (0.16)	22.74 (21.04, 24.45)	*P*
Ectopia cordis (10014144)	1	58.93 (6.88, 504.44)	58.93 (56.78, 61.08, 11.38)	0.97 (-0.12)	49.27 (47.48, 51.07)	*P*
Cardiac malposition (10007585)	1	36.83 (4.61, 294.50)	36.83 (34.75, 38.91, 7.27)	0.95 (0.04)	32.85 (31.11, 34.59)	*P*
Mitral valve atresia (10066800)	1	15.51 (2.08, 115.85)	15.51 (13.50, 17.52, 2.77)	0.9 (0.27)	14.78 (13.10, 16.47)	*P*
Congenital tricuspid valve atresia (10049767)	1	5.17 (0.72, 37.33)	5.17 (3.19, 7.15, 0.47)	0.74 (0.36)	5.1 (3.44, 6.75)	*P*
Charge syndrome (10064063)	1	32.74 (4.15, 258.43)	32.74 (30.67, 34.80, 6.45)	0.95 (0.08)	29.56 (27.84, 31.29)	*P*
Right aortic arch (10067407)	1	4.68 (0.65, 33.72)	4.68 (2.70, 6.65, 0.37)	0.71 (0.36)	4.62 (2.97, 6.27)	*P*
Congenital aortic valve incompetence (10010370)	1	4.53 (0.63, 32.67)	4.53 (2.56, 6.51, 0.34)	0.71 (0.35)	4.48 (2.83, 6.13)	*P*

RETRACTED

**Table 4:** Clinical indication of sertraline.

Characteristics	Reports, no. *n* (%)	
Indication	689	
Depression (10012378)	355	(51.52%)
Anxiety (10002855)	136	(19.74%)
Affective disorder (10001443)	71	(10.3%)
Product used for unknown indication (10070592)	24	(3.48%)
Perinatal depression (10078366)	15	(2.18%)
Ill-defined disorder (10061520)	11	(1.6%)
Panic disorder (10033666)	10	(1.45%)
Prophylaxis of neural tube defect (10054930)	7	(1.02%)
Adrenal disorder (10001347)	6	(0.87%)
Anxiety disorder (10057666)	6	(0.87%)
Morning sickness (10027975)	6	(0.87%)
Depressive symptom (10054089)	5	(0.73%)
Obsessive-compulsive disorder (10029898)	5	(0.73%)
Prophylaxis (10036898)	4	(0.58%)
Bacterial test positive (10059421)	3	(0.44%)
Generalised anxiety disorder (10018075)	3	(0.44%)
Major depression (10057840)	3	(0.44%)
Posttraumatic stress disorder (10036316)	3	(0.44%)
Psychiatric symptom (10061472)	3	(0.44%)
Bronchitis (10006451)	2	(0.29%)
Maternal drugs affecting fetus (10026923)	2	(0.29%)
Panic attack (10033664)	2	(0.29%)
Antidepressant therapy (10054976)	1	(0.15%)
Depressed mood (10012374)	1	(0.15%)
Disability (10013050)	1	(0.15%)
Maternal exposure timing unspecified (10071415)	1	(0.15%)
Mood swings (10027951)	1	(0.15%)
Nervous system disorder (10029202)	1	(0.15%)

RETRACTED

**Table 5:** Age and gender of top 20 adverse reactions associated with using sertraline.

	*n*	Gender						
		Average (month)	Male (*n*, %)		Female (*n*, %)		Unknown (*n*, %)	
Atrial septal defect (10003664)	146	5.43	61	(41.78%)	78	(53.42%)	7	(4.79%)
Heart disease congenital (10019273)	128	9.20	45	(35.16%)	43	(33.59%)	40	(31.25%)
Ventricular septal defect (10047298)	111	9.28	36	(32.43%)	63	(56.76%)	12	(10.81%)
Patent ductus arteriosus (10034130)	83	3.44	34	(40.96%)	44	(53.01%)	5	(6.02%)
Persistent fetal circulation (10034708)	34	1.00	18	(52.94%)	12	(35.29%)	4	(11.76%)
Fallot's tetralogy (10016193)	32	1.67	11	(34.38%)	16	(50%)	5	(15.63%)
Transposition of the great vessels (10044443)	31	3.75	14	(45.16%)	12	(38.71%)	5	(16.13%)
Pulmonary valve stenosis congenital (10037451)	21	0.00	6	(28.57%)	10	(47.62%)	5	(23.81%)
Cardiac septal defect (10064021)	21	0.00	3	(14.29%)	3	(14.29%)	15	(71.43%)
Pulmonary artery stenosis congenital (10037339)	21	2.50	8	(38.1%)	12	(57.14%)	1	(4.76%)
Coarctation of the aorta (10009807)	20	11.50	12	(60%)	6	(30%)	2	(10%)
Hypoplastic left heart syndrome (10021076)	19	6.33	14	(73.68%)	5	(26.32%)	0	(0%)
Bicuspid aortic valve (10004552)	17	9.33	11	(64.71%)	6	(35.29%)	0	(0%)
Congenital cardiovascular anomaly (10061054)	17	4.00	2	(11.76%)	4	(23.53%)	11	(64.71%)
Newborn persistent pulmonary hypertension (10053592)	15	1.00	9	(60%)	6	(40%)	0	(0%)
Haemangioma congenital (10018818)	14	1.00	11	(78.57%)	1	(7.14%)	2	(14.29%)
Congenital heart valve disorder (10064086)	12	10.50	9	(75%)	3	(25%)	0	(0%)
Pulmonary artery atresia (10037337)	10	21.00	6	(60%)	2	(20%)	2	(20%)
Congenital coronary artery malformation (10061060)	9	4.00	5	(55.56%)	4	(44.44%)	0	(0%)
Congenital aortic valve stenosis (10010371)	9	2.00	6	(66.67%)	2	(22.22%)	1	(11.11%)
Hypertrophic cardiomyopathy (10020871)	9	0.00	6	(66.67%)	2	(22.22%)	1	(11.11%)
Trisomy 21 (10044688)	8	1.00	3	(37.5%)	3	(37.5%)	2	(25%)
Double outlet right ventricle (10013611)	8	20.00	6	(75%)	0	(0%)	2	(25%)
Shone complex (10066802)	6	0.00	0	(0%)	6	(100%)	0	(0%)
Aorta hypoplasia (10049209)	6	4.00	3	(50%)	1	(16.67%)	2	(33.33%)
Atrioventricular septal defect (10063836)	5	2.00	1	(20%)	4	(80%)	0	(0%)
Ventricular hypoplasia (10047296)	5	1.00	4	(80%)	1	(20%)	0	(0%)
Congenital pulmonary artery anomaly (10061074)	5	5.33	2	(40%)	3	(60%)	0	(0%)
Multiple cardiac defects (10028178)	5	19.00	2	(40%)	2	(40%)	1	(20%)
Congenital mitral valve stenosis (10010548)	5	12.00	2	(40%)	2	(40%)	1	(20%)

## Data Availability

The datasets used and/or analyzed during the present study are available from the corresponding author on reasonable request.
